# Classification of Breast Cancer Images by Implementing Improved DCNN with Artificial Fish School Model

**DOI:** 10.1155/2022/6785707

**Published:** 2022-02-22

**Authors:** M Thilagaraj, N. Arunkumar, Petchinathan Govindan

**Affiliations:** ^1^Department of Electronics and Instrumentation Engineering, Karpagam College of Engineering, Coimbatore, India; ^2^Department of Biomedical Engineering, Rathinam Technical Campus, Coimbatore, India; ^3^Ethiopian Technical University, Addis Ababa, Ethiopia

## Abstract

Breast cancer is an important factor affecting human health. This issue has various diagnosis process which were evolved such as mammography, fine needle aspirate, and surgical biopsy. These techniques use pathological breast cancer images for diagnosis. Breast cancer surgery allows the forensic doctor to histologist to access the microscopic level of breast tissues. The conventional method uses an optimized radial basis neural network using a cuckoo search algorithm. Existing radial basis neural network techniques utilized feature extraction and reduction parts separately. It is proposed that it overcomes the CNN approach for all the feature extraction and classification process to reduce time complexity. In this proposed method, a convolutional neural network is proposed based on an artificial fish school algorithm. The breast cancer image dataset is taken from cancer imaging archives. In the preprocessing step of classification, the breast cancer image is filtered with the support of a wiener filter for classification. The convolutional neural network has set the intense data of an image and is used to remove the features. After executing the extraction procedure, the reduction process is performed to speed up the train and test data processing. Here, the artificial fish school optimization algorithm is utilized to give the direct training data to the deep convolutional neural network. The extraction, reduction, and classification of features are utilized in the single deep convolutional neural network process. In this process, the optimization technique helps to decrease the error rate and increases the performance efficiency by finding the number of epochs and training images to the Deep CNN. In this system, the normal, benign, and malignant tissues are predicted. By comparing the existing RBF technique with the cuckoo search algorithm, the presented model attains the outcome in the way of sensitivity, accuracy, specificity, F1 score, and recall.

## 1. Introduction

The most common disease for women is breast cancer. It is cells with extra growth of mass in women's breast region. This breast tissue forms the tumor, which is classified as benign or malignant. The malignant is the most affected cancerous region, and the benign is the non-cancerous region. This disease is diagnosed by biopsy. The researchers analyze various automated diagnosis approaches to determine breast cancer. The stroma maturity of cancer in the breast is classified by the histological image [1]. The breast cancer image of the stroma is the matured result of classification. Thermograph and mammography images are used for this approach. The thermograph images are taken from cameras, which are analyzed by infrared radiation and its intensity level. By comparing with the thermograph and mammogram, the mammogram image provides the exact result. The breast cancer images are classified using various machine learning techniques and artificial swarm optimization techniques. A capsule network model is performed in the preprocessing stage of breast cancer classifications [2].

The support vector machine learning, extreme learning machine, RBNN, DNN, and other classifiers performed the classification [3]. The optimization algorithms include ant colony optimization, honeybee optimization, PSO, genetic algorithm, and other artificial swarm intelligence techniques. The image processing methods are determined to classify the breast cancer images. The initial stage of classification in the image processing technique is the preprocessing step, which extracts the edges, filters the image, and improves the image quality. In medical image classification, feature extraction is the major procedure, and it gives data about the filtered picture. The feature selection process is carried out with bioinspired techniques. The classification supports various machine-learning approaches and deep learning techniques [4]. It classifies the normal, benign, and malignant properties of a given medical image. Biomedical images are used for disease classification. The images are ultrasounds, X-rays, computer-aided tomography, MRI, and other images.

In this, the CS optimizer is utilized for the selection process. The RBNN performs the characterization of the given image, which classifies the various properties from the input image [5]. Computer-aided diagnosis approach is a widely used technique for classifying the breast cancer image. It provides valuable information, and it utilizes general image classification techniques. The sampling process is used in the convolutional neural network for solving the computational complexity [6]. The sampling process is carried out in the pooling layer, which is performed with the neurons in the network layer. The LSTM structure is used for data analysis in CNN. An SVM learning technique is integrated with the decision-making algorithm for big data analysis [7]. The histopathological image is utilized to perform the classification and measures various performance metrics for analyzing the classifier. KM clustering approach and the SVM classifier with softmax techniques are utilized for modeling the classifier for medical imaging. The fuzzy-based entropy segmentation of the image processing method is optimized with the fish school algorithm [8]. Various grouping techniques use the artificial fish-school optimization algorithm. The conventional methods use a weka processor for breast cancer analysis [9]. The breast cancer image is used as either mammography or a histological image. This database is analyzed [10]. Computer-aided diagnosis technology is used for detecting breast cancer from images [11]. The CAD system improves the performance of breast classifications such as a benign, lesion, and malignant properties. Here, this tool is assisted by the radiologists in the mammographic screening process. In this, the morphological and texture feature extractions are performed in the segmentation approach [12]. Digital breast tomosynthesis is the three-dimensional image processing modality, which is developed with mammography and histological images. Based on the gradient field analysis, the true mass is measured for 3D images. The lesion property of breast cancer is analyzed using CAD technology. The softmax and ReLu function performance is performed in the CNN for breast cancer classification. The breast cancer dataset is available in open source, and it studies the breast cancer classification problems. The database has 7,909 samples with different classes. In these classes, benign and malignant are the most important properties. The 1024 × 1024 pixels of breast cancer images are taken for this proposed analysis. The training process in CNN uses the stochastic gradient descent technique.

The image augmentation process has different properties performed with various classes in the morphological approach. This image augmentation process performs the cropping, image resizing, enhancing, and random patches. Reference [13] has presented the DCNN for the classification model of breast cancer with the IRR approach. The pooling layer of the convolutional neural network reduces the spatial image size, and it performs downsampling. Based on the width and height of the image, the pooling layer gets a maximum pixel value of the image. The bioinspired techniques are applied in the image processing technique, especially to the classification approach. The bioinspired technique used for the application of breast cancer classification is ant colony optimization, genetic algorithm, PSO, etc. These methods improve the performance of feature selection. This optimization technique reduces the problem of overfitting and multiclass problem [14].

In the machine learning approach, the multilayer preceptor and the SVM are performed with two layers of the training process [15]. This approach uses the sequential minimal optimization algorithm, which depends on the performance of *c*, which means fuzzy logic. In the training process, the fuzzy rule is set for performing the feature extraction. The Kernel function is used to enhance the support vector machine learning technique. The k-means scheme is used in the feature extraction process. GLCM provides the result of energy, entropy, correlation, contrast, and homogeneity in the feature extraction process [16]. The breast cancer classification uses the machine learning technique [17]. The tissue detection, prognostic, and diagnostic are performed with different characteristics. The cross-validation technique is the important process used for partitioning the training and testing function [14]. The RBFNN is used for the flood forecasting technique, which is improved with the cuckoo search algorithm. The performance of the polyharmonic function has lesser error compared to the Gaussian approach. The deep learning technique is integrated to enhance the performance of CNN, which optimizes with the swarm intelligence approach [18]. The input layer of CNN takes the operation of preprocessing. The hidden layer analyses the feature of the given breast cancer images and the completion of pooling layer performance. The fully connected layer in the CNN will act to provide the output function. The direct preprocessed images are taken to separate the various properties of breast cancer. Based on the capsule network layer, the classification performance is worked. In this presented model, the CNN-based artificial fish school model is utilized for the classification of images in an enhanced manner. The normal, benign, and malignant are classified with optimum results. Here, this proposed method improves the accuracy, sensitivity, and specificity. The proposed image classification technique is used for various medical image processing and analyzing methods, and it gives the best result as compared with the existing work.

## 2. Literature Survey

Reis et al. [1] presented an automated image classification approach in the application of breast cancer analysis. The tumor tissue is classified into different classes. Here, the hematoxylin and eosin patterns are analyzed with the pathologist approach. The breast cancer prognostic method uses the normal picture, and local binary patterns are integrated with the RFC tree approach. Based on the tumor grade, the degrees are arranged with different types of breast cancer. Invasive breast carcinoma is the common breast cancer type, which mostly affects ladies. Mature, immature, and intermediate categories are analyzed in the stroma tissues. An ROI selection process is based on the input database, and it traces with randomly paired ROI. This provides the simultaneous result to observe the training and testing approach. The feature vector provides mature and immature properties. Here, the single-scale and multiscale properties are analyzed with mature and immature features.

Reference [2] illustrated the characterization of breast cancer images in the capsule network model. Here, the preprocessed breast cancer image with a histological property is used. The classification utilizes various systems such as ResNset, InceptNet, and AlexNet. These models are enhanced with the capsule network model, which classifies the breast image. It takes the direct preprocessed image for classification. In this approach, the benign, normal, in-situ, and invasive cancer type are classified. The stain normalization is the property of a patch reduction approach, which is used to avoid adverse effects on the staining. The input layer of the convolution type is created to perform the preprocessing stage. The capsule layer has primary and secondary sections for dimensional reduction. The dense layer is performed in the classification process. Here, the parameters are tuned to get the best preprocessed image for classification. The accuracy of both train and test layers is measured and compared with the conventional technique. Iteration range is increased for accuracy and loss prediction.

Reference [13] presented the convolutional neural network model for breast cancer. The inception recurrent residual network model is used in the CNN to characterize the image. Here, the DL approaches with CNN; it gives the robust execution with inception and residual networks. Here, the BreakHis dataset is used for classification. In the preprocessing stage, the original image improves the quality by resizing, removing noise, image augmentation, and patching. After that, it performs the feature extraction process. Finally, it performs the feature selection process. The limitation of this technique is the design complexity. The results are measured to analyze with various conventional methods. The accuracy, ROC, AUC, and global accuracy are calculated, and they classify different types of benign and malignant features.

Reis et al. [1] have introduced the classification technique and used the bioinspired techniques. Here, various machine learning approaches are modeled to separate breast cancer, and the optimization technique is used in the feature selection process. The image types such as the histological image, pathological, and thermography images are used for breast cancer classifications. Hence, the SVM technique is utilized for classification, and it is compared with utilizing different bioinspired optimization techniques, that is ACO and PSO. Initially, the thermography images are applied for the preprocessing stage, which is performed with grey-scale imaging, and it reduces the noise since it improves the input image quality. The feature extraction process used the GLCM process. The feature selection technique utilizes bioinspired techniques such as ACO and PSO. Finally, it results in the classification using SVM. The accuracy, sensitivity, specificity, and recognition time are measured to obtain the resultant parameter.

Reference [3] analyzed the machine learning approach for classifying breast cancer images. Here, the machine learning scheme is used as a classifier, and it optimizes the Bayesian classifier. This method is utilized to identify and prognostic the breast cancer tissues. Here, the binary classification scheme is applied in the Bayesian classifier. In the preprocessing stage, the edges are removed to enhance the image quality. The feature extraction process is carried out with KNN, and it also performs the clustering. This approach finds different classes in the testing and training procedure. It helps to separate the features of the image. The reduction approach is employed to select different features, and it uses the cross-validation technique. The precision of both training and testing is calculated to compare with the existing work. Without using the optimization technique, it makes the reduction process inefficiency.

Reference [19] proposed the artificial fish school optimization algorithm for the grouping approach. The common method of grouping strategy is the deterministic finite automaton technique. However, it searches only the local environment since the artificial fish-school optimization approach is used, and it is used for global search. The grouping strategy uses the heuristic algorithm with intelligent optimization. The behavior of the artificial fish is used for the global optimization technique. The encoding process is grouped with the 2D array model, and it is represented with the different group expressions. The interaction rate of the artificial fish is used for the grouping algorithm. The increased amount of food in the area is searched by prey behavior. The drawback of grouping is reduced by the behavior of the swarm. The random search movement is selected by a fish interaction rate. By comparing with other optimization algorithms such as PSO, ACO, and GA, the artificial school optimization algorithm achieves the result.

Reis et al. [1] have described the optimization technique for performing the training process in the DCNN. Here, the swarm intelligence technique is used for optimizing the training process of the DCNN. Here, this optimization technique uses the artificial fish school optimization algorithm. In this approach, the text patterns are used as a dataset. This text mining process is analyzed with a random search. This text mining approach is also applicable for various statistical data science tasks. The vector optimization is performed by using FSS. The preprocessing of input text uses word2vec, and the final layer of CNN provides the statistical information. After performing training and testing, the precision of the text-mining task is calculated to obtain the result. The technique performs the maxpooling and softmax in the feature extraction process of CNN, and it normalizes the functions by splitting the classes. The text is trained to provide the vector output, and it is optimized using FSS. Then, it performs testing to predict the accuracy.

Reference [20] presented the artificial fish school optimization technique for optimizing the functions. Here, the global optimum value is selected for function optimization. This method is compared with GA, ACO, and PSO. The function optimization task is performed by selecting the functions from search space. After selecting the functions, the AFS initializes the population, distance, max iteration, and crowding factor. The population initialization gives the exact integer space. The bulletin initialization has calculated the present state of fish, and it selects the best behavior of fish. To update the bulletin simulations, the met condition is used to select the best behavior of AF. The process is terminated after obtaining the optimum solution with optimum values. The accuracy and computation time are calculated and compared with the conventional techniques.

Reference [4] presented the breast cancer classification scheme and used the deep learning approach. The multilayer perceptron algorithm is used to calculate the best accuracy. The feature extraction and reduction are performed in the deep neural network model. Ten attributes are used in two different classes, and it is classified with the inbuilt process of the deep neural network. The 8-fold and 10-fold cross-validation technique is performed in the multilayer perceptron algorithm. In this paper, the dataset is collected from the oncology department at Medical Centre University, Yugoslavia. These datasets are not a label but a random dataset. Based on the weight of the neurons, the MLP is performed with the mathematical activation function. Weka 3.8 is utilized for the classification of breast cancer. After performing the cross-validation scheme, the precision of each scheme is calculated.

Reference [5] introduced the classification scheme for cancer images. Here, the back propagations NN and RBNN are used as a classifier. In this paper, the feature extraction process has a significant role in the classification approach, which utilizes the grey-level co-occurrence matrix. The MIAS database is utilized for the classification approach. The initial stage of classification detects either normal or abnormal. If it is abnormal, the next stage predicts either malignant or benign. The GLCM process extracts features such as correlation, entropy, homogeneity, and variance. By comparing both RBFNN and BPNN, the radial basis neural network achieves the classification results. Accuracy and mean squared error are calculated to achieve the result.

Reference [9] described breast cancer analysis. This process is carried out by performing with WEKA. The proposed work performed a sJ48 classifier, which gives the best accuracy result. During preprocessing, the missing traits are neglected. The classifiers performed in this paper are J48, REP Tree, and Naïve Bayes. Here, K-means clustering and farthest first clustering methods are employed to reduce the complexity in the feature extraction procedure. The number of classified instance with correctness and incorrectness is measured for three classifiers. The accuracy and computation time give enhancement in the three classifiers. The WEKA programmer is used with the machine learning approach for classifying breast cancer.

Reference [8] presented the image segmentation model using the fuzzy entropy technique, which is segmented by the artificial fish school optimization algorithm. Here, the maximum entropy level is selected by the fuzzy rule, and it is used for image segmentation. The histogram images are used to process with the segmentation process. Here, the threshold technique is used to optimize the result through Otsu's threshold model. The maximum entropy is achieved by the threshold algorithm. The AFS algorithm is used to optimize the parameter from the entropy algorithm. In AFS, each fish behavior is evaluated to get the objective function. The image segmentation is performed with the fuzzy entropy model. Here, the double threshold-based image segmentation method improves the entropy level using fuzzy rules. The tire image is taken to perform the image segmentation. The fuzzy entropy level is obtained for both GA and AFS. Here, the optimization performs foraging, clustering, and tailgating.

Reference [21] presented a deep learning technique. This process is developed to improve breast cancer risk prediction. The breast cancer database is taken from a larger tertiary academic medical centre. The mammograms are filtered to analyze the function. The dataset is validated to analyze the data. Based on the patient information (attributes), the cancer set and dataset are separated by examining training, validating, and testing. The hazard ratio and position of the top/bottom decile flow are measured. The hypothesis model has mammography information to capture the cancer-risk state. The Tyrer-Cuzick version is used for hybrid deep learning. Here, the confusion matrix analyzes the density factor of the breast cancer image.

Reference [10] described about the breast cancer dataset for histopathological image classifications. The medical image classification is performed with the automated classification using a computer-aided diagnosis tool. Here, the two classes are used to compute the breast cancer region. ML scheme is modeled to utilize the classification of the medical image. The BreaKHis dataset is taken to test the classification of the breast cancer image model. Malignant and benign image sets are classified with different properties. A completed local binary pattern is utilized in the extraction process, and the texture feature is extracted by the GLCM process. The surf and sift are detected using the oriented fast and rotated brief process. Four different classifiers are used with various feature extraction approaches. Reference [14] utilized the GCNN and CNN for breast cancer classification.

## 3. Proposed Method

The proposed Deep CNN for classifying the breast cancer image is optimized using the artificial fish school optimization algorithm and is modeled to provide the best classification result. In this section, the proposed methodology is described with classifier and optimization technique and their application of breast cancer image analysis.

### 3.1. Deep CNN Using AFS Optimization for Classification

Here, the artificial fish school technique is used to give the direct image set to the training process of the classifier. The random permutation of the AFS is selected by initializing the direct values. The maximum epochs are given in the optimizer at the stage of variable initialization. Hence, the preprocessing stage is performed with the wiener filter for improving the quality of the image. These filtered images are sent to the convolution layer, which sets the image to filter with a convolution filter for activating the features of the given breast image. The convolution 2D layer will normalize the image to perform the training process in the ReLu layer. The pooling layer selects the higher value of the image by the sampling process. The single GPU processor is used for Deep CNN to perform classification. The AFS algorithm provides a direct training image to the Deep CNN. Based on the training image, the supposition accuracy is given in the AFS. The convolution neural network having three layers with sublayers is used. The activation function enables the feature map for the regional size of each image. Then, it sends to the pooling layer for selecting the maximum value of the trained image. The proposed Deep CNN architecture is given in Figure 1.

In the convolution neural network, the above-mentioned layers performed different functions to activate the process. In this proposed method, the 90 input images are extracted for classifying breast cancer, which is given to the input layer of CNN. It is normalized in this convolution layer. The MIAS dataset is extracted for breast cancer images, and it has 1024 × 1024 pixels. A single GPU processor is capable to analyze the 64 × 64 image pixels since it is resized to perform the feature extraction. The convolution 2D layer is processed with the grey-scale image of breast cancer image to remove the features.

Here, the ReLu layer is used to provide the positive images to the CNN; otherwise, it outputs to zero. The pooling layer is the major function to activate the CNN. Here, the greater pooling layer is utilized to select the maximum value of pictures from the ReLu layer. The fully connected layer gives the output of feature extraction by classifying the breast cancer image. The extraction procedure is activated in the pooling layer. The probability of picture is applied in the multiclass functions, and it is performed with the softmax layer. In this, the artificial fish school optimization algorithm is implemented for selecting the training image with supposition accuracy. A single Deep CNN process performs the three operations such as feature extraction, feature selection, and classification. The accuracy, sensitivity, specificity, and computation time are measured to analyze the performance.

#### 3.1.1. Dataset

The MIAS database is utilized to separate the images of breast cancer from mammography. The database is downloaded from http://peipa.essex.ac.uk/info/mias.html. The mammographic picture analysis society provides the digital mammogram image for classifying the different features. The database comprises of seven columns representing image, type of tissue, abnormality, its size, location, stage, and image information. This classification approach is also capable to analyze the screening mammography with a digital database. In this proposed system, the MIAS database is used, which has 200-micron pixel with the padding of 1024 × 1024. The dataset containing 322 digits with 2.3 GB 8 mm tapes is used. This digital mammogram has the density of 0–3.2, and it is represented with each single pixel that has 8 bits. The MIAS database has different characters of background tissues. The abnormality of the breast cancer image is classed by masses, image distortions, asymmetry, and calcification. It classifies malignant, benign, and normal breast images.

#### 3.1.2. Preprocessing Stage

The first stage of mammography image classification uses the preprocessing step to enhance the image quality. The input has 1024 × 1024 pixel size, which is resized with 64 × 64 pixels. The wiener filter is used in this preprocessing stage. The 2D convolution operation removes the noise presented in the input signal. The overlapping patches, removing edges, improving the visual quality by removing the noise, resizing, and filtering are performed in this process. Here, the normal, benign, and malignant images are filtered using the wiener filter.

#### 3.1.3. Deep CNN

The CNN is the type of a deep learning technique. The DNN model performs the same operation in the convolutional neural network. The proposed Deep CNN is modeled to separate the breast cancer image with the characteristics of normal, benign, and malignant. This process performed with various layers of convolution approach is as follows:

(i) Convolution 2D layer: this layer is used for normalizing the input pictures to perform the feature extraction process. The 2D convolution process involves the operation as follows:
  (1) $$\begin{array}{c} f1\left(\text{Ps}\right)=\max\left(0,\text{weignt}*P+\text{BF }1\right),\\ f\left[u,v\right]*g\left[u,v\right]=\sum_{n=-\infty }^{+\infty }\sum_{m=-\infty }^{+\infty }f\left[n,m\right].g\left[u-n,\;v-m\right]\;. \end{array}$$
(ii) This process improves the image by the normalizing factor. This allows the 2D matrix images for normalizing the values. This performance is done with the grey scale image.
(iii) Rectified linear unit layer: the ReLu layer activates the neurons presented in the convolutional neural network. It selects the maximum value in the function of *f*(0, *x*). It acts as a rectifier, and it performs the differentiations by neuron points in the network. Feature representation with prefiltered images is represented as follows:
  (2) $$\begin{array}{c} f2\left(\text{Ps}\right)=\text{max}\left(0,\text{weight}*f1\left(\text{PS}\right)+\text{BF }2\right). \end{array}$$
  (3) $$\begin{array}{c} P\left(v=\text{ki}|u,g,{\text{weight}}_{i}\right)=\;\frac{e^{\text{gk}\left(u,\text{wk}\right)}}{\sum_{i}^{k}e^{\text{gk}\left(u,\text{wk}\right)}}. \end{array}$$
(iv) The nonlinear rectification is performed to activate CNN functions. The nonlinear function activation is the major concern for various systems. The probability function with different classes is given as follows:
(v) Max. Pooling layer: the pooling layer is employed to perform the feature extraction process. Here, it selects the maximum value of breast image to activate the pooling layer. The training image sets are selected randomly from the artificial fish-school optimization technique. It also assumes the accuracy of the each image sets.
  (4) $$\begin{array}{c} f3\left(\text{Ps}\right)=\text{max}\left(0,\text{weight}*f2\left(\text{Ps}\right)+\text{BF }3\right). \end{array}$$
  (5) $$\begin{array}{c} L=-\overset{l}{\underset{i=1}{\sum }}\ln\left(P\left(v=\text{ki}|u;g;\text{weight}\right)\right)=\;\overset{l}{\underset{i=1}{\sum }}\ln\left(\sum_{i}^{k}e^{\text{gk}\left(u,\text{wk}\right)}\right)-g_{v^{i}}. \end{array}$$
(vi) The objective function with maximum value representation is given by
(vii) The spatial size of the image is reduced for the feature reduction approach. It operates only with the feature map of each image. The maximum subsampling of the pooling layer will map the features based on the classes. The 3x3-convolution matrix strides are used to select the maximum value. The selected training dataset is labeled with the different classes, and it performs testing. Based on the stride and padding in the matrix, the ReLu performs to activate the pooling operation.
(viii) Fully connected layer: it is the output of feature maps, and it is performed with the AFS optimization. Each node in the Deep CNN is interconnected to perform the breast cancer image classification. It performs the feed-forward neural network model by connecting the feature reduction approaches in the convolution layer. It holds the information about the image features and provides in the vector form. The pooling layer reduces the feature map, and it is optimized with the AFS algorithm, which is connected to perform the classification. The training process selects 22 images, and the testing process is carried out with 8 images. Here, the epoch is 20 based on this; the training process will be performed to provide the classification accuracy.
(ix) Softmax layer: the softmax layer solves the multiclass problems of integral functions. It selects the maximum value of final class predictions. The softmax activation function normalizes the input image and provides a positive result. The nodes of the fully connected layer are the softmax layer, which activates the function by selecting the multiclass classifications. The pretrained set of images is configured with the dense characteristics of a given dataset.
(x) Classification layer: the classification layer is the output layer of the Deep CNN, and it provides the classified result of breast cancer images. It has the functionality to know about the image features. Based on stride representation, image pixels are shifted to the matrix. Then, it performs the feature extraction and reduction using Deep CNN layers. The Deep CNN layers form the array in the order of the above-mentioned layers.

(6) $$\begin{array}{c} \text{output}=\text{sigmoid}\left(L\right). \end{array}$$

#### 3.1.4. Artificial Fish School Optimization Algorithm

The optimization of image classification is an important process. In this proposed method, the artificial fish school optimization algorithm is employed to provide the direct training files to the classifier. It also gives the approximate accuracy for each training image. Initially, the population size, crowding factor, maximum iteration, and distance are given in the parameter initialization process. Then, the population is initialized to produce the weight of the fish. The bulletin initialization process evaluates the present state of fishes. If the state of best fish and its position is found, it terminates the process; otherwise, it again performs the operation to select the best AF.

  Requires Deep CNN Output Vector of feature map
(1) For *i* *=* 1 to *Number of Epoch* Do
(2) Start
(3) Initialize *location*
(4) Initialize the *crowd of the fish*
(5) Evaluate *fitness*
(6) While
(7) *no of epoch* is not obtained
(8) Do
(9) Analyze the *unique movement*
(10) Calculate the *fitness*
(11) Enhance the *new location*
(12) Analyze the *fitness difference*
(13) Analyze the *fish weight*
(14) Analyze the *variance of the weights*
(15) Analyze the *instinctive movement*
(16) Enhance the *new location*
(17) Analyze the *barycentre*
(18) Analyze the *volitive movement*
(19) Evaluate the *fitness*
(20) Enhance the *individual step*
(21) Update the *volitive step*
(22) End For

In the presented model, the AFS algorithm is implemented to select the training image, and it provides directly to the image classifier. It also provides the respective accuracy to the images. This optimal solution is used to train the image, and it is tested. These images are classified based on the features. The approximate accuracy is used for the classification result. The training accuracy is approximately given to the Deep CNN. However, it is not an exact accuracy result of the classifier. The objective function of AFS is given by

(7) $$\begin{array}{c} X_{a}=X_{b}+\text{training data}\left(n\right). \end{array}$$

The artificial fish performs swarming that is given in the following expression:

(8) $$\begin{array}{c} X_{b}^{m+1}=X_{b}^{m}+\;\frac{X-X_{b}^{m}}{\left|\left|X-X_{b}^{m}\right|\right|}.\text{train data}\left(n\right). \end{array}$$

If the artificial fish follows the neighbor partners for food search, the behavioral description represents the fitness value. The forward companion of AF while getting the fitness value is given by

(9) $$\begin{array}{c} X_{a}^{m+1}=X_{a}^{m}+\frac{X_{b}-X_{a}^{m}}{\left|\left|X_{b}-X_{a}^{m}\right|\right|}.\text{step }.\text{ train}\left(n\right). \end{array}$$

The movement of the AF selects the path randomly, and its prey behavior is given by

(10) $$\begin{array}{c} X_{a}^{\left(m+1\right)}=X_{a}^{m}+\text{visual }.\text{ random}\left(n\right). \end{array}$$

The best possible image is selected by the following equations:

(11) $$\begin{array}{c} \text{if}\left(\text{Best AF}\left(k\right)-\text{Best AF}\left(l\right)\right)<\text{iteration},\\ X_{\text{some}}^{m+1}=X_{\text{some}}^{m}+\beta .\text{visual }.\text{ random}\left(n\right),\\ X_{a}^{m+1}=\;X_{a}^{m}+\left(\frac{X_{b}-X_{b}^{m}}{\left|\left|X_{b}-X_{b}^{m}\right|\right|}+\frac{X_{\text{bestAF}}-X_{a}^{m}}{\left|\left|X_{\text{bestAF}}-X_{a}^{m}\right|\right|}\right)*\text{AF}\_\text{step}*\text{random}\left(n\right),\\ X_{a}^{m+1}=X_{a}^{m}+\text{AF}\_\text{visual}*\text{random}\left(n\right). \end{array}$$

The global search of the AFS algorithm is to optimize the training image to perform classification. The convergence speed shows the search optimization result of AF. Artificial fish school optimizer finds better classification accuracy. In this proposed image classification method, the convolution layers performs the extraction and reduction procedure, which is optimized by selecting the direct training files to the classifier. This optimization algorithm performs the behavior of the artificial fish to select the food in the sea. This scheme is applied to the CNN for direct selection of training images. The sensitivity, accuracy, and specificity of the proposed scheme are analyzed to compare with the existing work. By this performance analysis, the accuracy, sensitivity, and specificity are achieved for the presented model.

## 4. Results and Discussion

Thus, the classification of breast cancer images using DCNN and AFS optimization algorithms is modeled, and it obtains the best outcome as compared to the previous work. The MIAS dataset helps to classify the images of breast cancer with three stages, that is, normal, benign, and malignant. These images have 1024 × 1024 pixels in size. The input data of normal breast cancer images are illustrated in Figure 2. The total input breast images in the information base are 90. For each property, it selects 30 sets of images to classify the normal, benign, and malignant tissues. For the first set, the Deep CNN takes 22 images to train the network. The testing process utilizes 8 images. Here, the input image of benign and malignant is shown in Figures 3 and 4, respectively. Initially, the preprocessing stage filters the input image using the wiener filter. A single GPU processor does not accept large size images since it is resized to 64 × 64 pixels.

The preprocessing stage of classification uses the wiener filter for resizing and filtering the breast image input. Here, 64 × 64 images are applied to DCNN for classification. The properties of the breast image are filtered with the help of the wiener filter, which is shown in Figure 5.

Here, the AFS optimization algorithm is used to select the training images while performing the feature extraction process in Deep CNN. The optimal result is found in the fifth position of the training set, and its average accuracy is provided.  Figure 6 shows the simulated result of the artificial fish school algorithm, which provides the best possible training set with respective average accuracy. The CNN layers perform various operations with respective functionalities. A single processor performs three sets of functionalities as extraction, reduction, and classifications. Hence, the result of CNN is shown in Figure 7. Here, various performances in the CNN result in the classifier efficiency.

The optimal training image position and its corresponding accuracy from AFS optimizer is shown in Figure 6.

The training process in Deep CNN uses the direct selection of the training file, which uses the artificial fish-school optimization process. Here, 20 iterations are performed to obtain the best result, and they also give the reduced losses of both training and testing. The training progress is shown in Figure 8.

In this, the proposed Deep CNN using AFS optimizer provides the best result, and its performance is evaluated (see Figure 9) based on the different classes assigned in the network. The confusion matrix arranges the TP, TN, FP, and FN ranges to analyze the accuracy, sensitivity, and specificity.

Performance evaluation parameters are calculated by obtaining the result of accuracy, recall, and F1 score. In this, accuracy, sensitivity, and specificity are calculated to achieve the result of overall performance of the Deep CNN using the AFS algorithm.

(12) $$\begin{array}{c} \%\text{ of accuracy}=\;\frac{\text{True Neg}+\text{True Pos}}{\text{True Pos}+\text{False Pos}+\text{False Neg}+\text{True Neg}}\;x\;100,\\ \text{sensitivity}=\frac{\text{True Pos}}{\text{True Pos}+\text{True Neg}},\\ \text{specificity}=\frac{\text{True Neg}}{\text{True Neg}+\text{False Pos}}. \end{array}$$

By this measurement, the performance is evaluated for both training and testing processes. The comparison result of proposed and existing methods is given in Table 1

Time complexity is the time required for running the process. In the proposed method, the time complexity is reduced with the minimal training images. In the presented work, the image classification is modeled based on the deep learning approach of the convolution neural network. This technique provides the classified result by optimizing the training process in the classifier, which uses the behavioral approach of the artificial fish-school optimization technique. The accuracy, sensitivity, specificity, and computation time of both training and testing processes are evaluated and compared with the conventional approach. The proposed Deep CNN using the artificial fish school model achieves the best result for breast image classifications. Therefore, the analysis report shows that the proposed Deep CNN using the artificial fish school is a better image classifier than the conventional methods.

## 5. Conclusion

The artificial fish-school optimization technique is used for selecting the number of epochs in the design of the deep convolutional neural network model, and it is utilized for classifying the mammography images from the MIAS database which is presented. It can classify the malignant, normal, and benign characteristics of breast cancer images. Here, the single CNN mode performs the three operations like preprocessing and feature extraction, and also it enhances the design model. The Deep CNN is optimized using AFS in the training process. Here, the artificial fish-school optimization technique selects the training images by directly assigning them to the classifier. Here, this optimizer also provides the average accuracy level of the training images. This enhancement makes the system efficient by a reduced computation time. Here, the proposed CNN model performs feature extraction, feature reduction, and classification. By comparing the performance analysis of the proposed method versus conventional methods, the proposed Deep CNN using AFS optimizes the result by providing better accuracy, sensitivity, and specificity. Thus, the system concludes that the breast image classification is performed efficiently using Deep CNN based on the AFS algorithm. In the future, the optimization technique is improved for utilizing the operations in both training and testing processes. The CNN model is modified to provide better efficiency than this system. These numbers of properties are extracted to characterize the various properties in breast cancer images. The proposed work is concentrated only on the training image and epoch. It can be improved by including other hyperparameters. [23–31].

## Figures and Tables

**Figure 1:** Architecture of the DCNN model.

**Figure 2:** Input image (normal).

**Figure 3:** Input image (benign).

**Figure 4:** Input image (malignant).

**Figure 5:** Filtered images. (a) Normal, (b) benign, and (c) malignant.

**Figure 6:** Result of AFS optimizer.

**Figure 7:** Simulated result of deep convolutional neural network.

**Figure 8:** Training progress in Deep CNN using AFS optimizer.

**Figure 9:** Performance evaluation of the proposed method.

**Table 1:** Comparison result of performance evaluation.

Parameters	Existing work [22]		RBFNN using CSO		Deep CNN using AFS	
	Training	Testing	Training	Testing	Training	Testing
% of accuracy	97.1	97.0	100	98.3	100	98.66
Sensitivity	0.96	0.96	100	0.98	100	0.991
Specificity	0.97	0.96	100	0.98	100	0.988
Computation time	55sec	30sec	52sec	30sec	20sec	16sec

## Data Availability

The data used to support the findings of this study are available from the corresponding author upon request.
